The article "The role of apatinib combined with paclitaxel (aluminum binding type) in platinum-resistant ovarian cancer" was retracted in 2021. Reasons: duplicated images; unreliable data.

# The role of apatinib combined with paclitaxel (aluminum binding type) in platinum-resistant ovarian cancer

**DOI:** 10.1186/s13048-020-00719-3

**Published:** 2020-09-21

**Authors:** Hong Zhao, Rong Li, Xiaoyan Wang, Xin Lu, Min Hu, Jinbin Zhang, Xia Zhao, Xiaoqin Song, Yangyang Liu

**Affiliations:** 1 Department of Biochemistry and Molecular Biology, Basic Medical College, Shanxi Medical University, No. 56 Xinjian South Road, Yingze District, Taiyuan City, Shanxi Province China; 2 Department of Gynecology, Shanxi Cancer Hospital, Taiyuan, China; 3 Shanxi province center for disease control and prevention, Taiyuan, China; 4 The Second Affiliated Hospital of Shanxi Medical University, Taiyuan, China

**Keywords:** Apatinib, Paclitaxel (aluminum binding type), Ovarian cancer, Combined medication

## Abstract

**Objective:**

To assess the anti-tumor activity and side effects of different dosages of paclitaxel (albumin binding type) (hereinafter referred to as nab-P) combined with Apatinib (hereinafter referred to as AP) in platinum-resistant ovarian cancer cell line and xenograft models.

**Methods:**

SKOV-3/DDP cell line was selected as the research object in cytology experiment. Firstly, we divided it into three groups for experiments to explore the individual effects of nab-P and AP. a): Control group, blank control, no drug intervention; b): nab-P group, nab-P 40 μmol/l; c): AP group, AP 50 μmol/l (Drug doses were IC-50 values that detected by MTT assay). Apoptosis related protein (Bax, bcl-2), vascular related protein(p-VEGFR-2), invasion related protein (MMP-2) expression were detected by Western blot and Cellular immunofluorescence, the invasion ability of tumor cells were detected by Transwell and Cell scratch test. Based on these dates, secondly, establishing different doses of nab-P combined with Ap to explore the curative effect of combination therapy. a): Control group, blank control, no drug intervention; b): Group-1, nab-P 5 μmol/l + AP 10 μmol/l, c): Group-2, nab-P 4.5 μmol/l + AP 10 μmol/l, d): Group-3, nab-P 4 μmol/l + AP 10 μmol/l, e): nab-P group, nab-P 5 μmol/l, f): AP group, AP 10 μmol/l (MTT assay). The combination index was analyzed by Compusyn software, Western blot, Immunofluescence, Transwell and Cell scratch test also were also chose to observe of inhibition effect. Thirdly, we used xenograft models to verify the results of cytological experiments. Tumor-forming BALB/c female nude mice were randomly divided into 4 groups, a): Control group, no drug intervention, only saline injection, b): nab-P 20 mg/kg + AP 150 mg/kg, c): nab-P 18 mg/kg + AP 150 mg/kg, d): nab-P 16 mg/kg + AP 150 mg/kg (The doses were guided by the pharmaceutical manufacturers). The tumor growth curve was analyzed during the experiment. And the apoptosis related protein (Bax, bcl-2), angiogenesis related protein (CD31, p-VEGFR-2) and invasion related protein (MMP-2) were observed by Western blot, Immunofluescence and Immunohistochemistry to analysis the ant-tumor effects. The quality of life in nude mice were observed to analysed the drug-induced side effects.

**Result:**

In the separate medication section, (1) The IC-50 value of nab-P was 45.53 ± 4.06 μmol/l, while the AP was 50.66 ± 4.96 umol/L (48 h). (2) The expressions of bcl-2 (nab-P group, AP group), p-VEGFR-2 (AP group), MMP-2(nab-P group, AP group) were higher than Control group, while Bax (nab-P group, AP group) lower (*P* < 0.01). (3) The cell invasive ability was decreased after the nab-P and AP intervation (P < 0.01). In the combination medication section, (1) Compusyn showed the Combination index (Cl) were all below 1 (Cl < 1), that means nab-P and AP are synergism. (2) The combination IC-50 value was nab-P 5.28 μmol/l + AP 10.56 μmol/l (48 h). (3) In the detection of related protein expression, the combination of drugs can improve the anti-tumor effect, otherwise, after combined with AP, when nab-P were reduced dose in proper quantity, there were no obvious different in drug effect. (4) After reducing the doses of nab-P, the average food intake of nude mice increased from 4.50 g ± 0.17 to 5.55 g ± 0.13, and the one-hour activity increased from 6.11 min ±0.16 to 6.34 min ±0.13.

**Conclusion:**

nab-P, a chemotherapeutic agent, can play an anti-tumor role in platinum-resistant ovarian cancer, but it can cause adverse effects that increase with dose. When combined with AP, the two drugs have synergistic effect, which can improve the anti-tumor effects of single drug. In addition, when combined with AP, the doses of nab-P can be appropriately reduced under the standard of recommended to reduce the toxicity of chemotherapy drugs, without affecting the anti-tumor effect.

## Introduction

Ovarian cancer (hereinafter referred to as OC) is one of the three common malignant tumors of female genital system, known as “silent killer”. Because OC is a high malignancy with insidious onset, invasive fast-growing, high recurrence rate and fatality, most patients have reached the late stage (stage III or IV) when they seek medical advice. According to the 2018 latest official statistics released by the international cancer research center, the number of morbidity and deaths from OC in the world is 295,000 and 185,000, respectively [1]. In the 2019 version, the National Comprehensive Cancer Network (NCCN) guides the first-line chemotherapies that are still represented by platinum. These drugs have a significant effect on the treatment of patients, with a five-year survival rate of 47% [2], but about 60% will recurrence unfortunately [3]. In addition, among these patients, most of these were platinum-resistant recurrence (platinum-free interval < 6 months). Platinum-resistant recurrent is an important factor that makes the patient’s condition difficult to control. There are studies have shown that more than 80% of patients with platinum-resistant recurrent had only 12–18 months for progression-free survival (PFS) [4]. More importantly, the number of patients who develop platinum-resistance are increasing, compared with 30–40% of OC patients with platinum-resistance in 2012 [5], the data in 2019 increased to 70–80% [6]. In response to the above phenomena, in clinic, most platinum-free drugs are chosen to improve the sensitivity of the patient itself, such as liposome adriamycin, nab-P and so on [7].

nab-P is based on paclitaxel, and human albumin is added as carrier and stabilizer, and the molecular weight is about 130 nm. It can be directionally adsorbed on the corresponding tumor cells by SPARC protein, and then kill them [8]. Compared with standard paclitaxel, it can increase the local cancentration of drugs, enhance the anti-tumor effect, and improve its own stability and safety. In 2005, a phase III clinical trial of breast cancer showed that nab-P was significantly more effective than standard paclitaxel (effective rates were 33 and 17%, respectively, *P* = 0.001) [9]. In other study of xenograft models of lung, ovarian, prostate and colon cancer, nab-P produced less drug toxicity than standard paclitaxel at the same dose [10]. In addition, nab-P also played a good synergistic effect in combination therapy, such as Volk’s research in breast cancer, combined with bevacizumab had gotten satisfactory results [11].

In recent years, the development of targeted anti-tumor drugs has promoted the precise treatment process of cancer. Tyrosine kinase (TK) is an important target only next to G protein-coupled receptor [12], and one study has shown that tyrosine kinase inhibitors (TKI) can increase the effect of chemotherapy drugs, mainly by inhibiting the function of ABC transporter [13]. Apatinib, a TKI-targeted drug, can highly selectively act on the ATP binding site of vascular endothelial growth factor receptor-2 (VEGFR-2), and then block the downstream phosphorylation of VEGFR-2 to inhibit tumor angiogenesis [14]. Many research have shown that AP has showed strong tumor inhibition and individual tolerance in non-small cell lung cancer, gastric cancer, breast cancer and other malignant solid tumors [15–17]. In OC, many achievements have also been made. In a phase II clinical study of recurrent epithelial ovarian cancer, the objective response rate (ORR) of patients was 41.4%, and PFS was 14.5 months [18]. In 2018, an article published in *Lancet Oncol* on the treatment of advanced ovarian cancer patients with AP and Etoposide showed that up to 54% of patients achieved remission [19], and in the same year, Jiuhuan [20] found that the combination of AP and standard paclitaxel can significantly inhibit tumor growth.

Therefore, we propose whether AP combined with nab-P can improve the therapeutic effect on OC patients. Moreover, because the recommended dosage of nab-P is 260 mg/m^2^, the use of large dosage aggravates the physiological burden of patients inevitably, we assumed that if we can reduce the dosage of nab-P without effecting the efficacy after combination with AP. This paper preliminarily discusses the antitumor effect of the combination of nab-P and AP in the treatment of OC, so as to provide reference for clinical medicine.

## Materials and methods

### Equipments and drugs

The equipments used in the experiment is as follows: Power Pac-TM Alkaline electrophoresis apparatus (164–5051, Bio-Rad), Gel imaging analysis system (SYNGENE G: BOXChemiXR5), Microplate Reader (Awareness Stat Fax, USA).

The drugs used in the experiment are as follows: Apatinib tablets (Jiangsu Hengrui Pharmaceutical Co., Ltd., Jiangsu, China, H20140103, 250 mg), paclitaxel (aluminum binding type) (Shiyao Holding Group Co., Ltd., Shijiazhuang, China, H20183318, 100 mg). Use after dissolving with Dimethyl Sulfoxide (DMSO, Sigma-Aldrich Co., St Louis, MO, USA).

### Cell lines and culture

SKOV-3/DDP cell line was purchased from Procell (Procell Life Science & Technology Co., Ltd., Wuhan, China), and identified by short tandem repeat (STR) analysis. The cell line was cultured in RPMI 1640 medium (Boster Biological Technology co,.Ltd., Wuhan, China), supplemented with 10% fetal bovine serum (Cellmax, Beijing, China), and incubated in 37 °C, 5% CO_2_ incubator.

### Cytotoxicity assay

The cytotoxicities of AP and nab-P for SKOV-3/DDP cell line were determined by MTT assay (Sigma-Aldrich Co., St Louis, MO, USA). Inoculate 1 × 10^4^ cells/well in 96 well cell cultrue cluster. The concentration range of nab-P were 5 × 10^− 2^ to 5 × 10^2^ μmol/l, and AP 10^− 1^ to 10^3^ μmol/l. In the experimental group, 100 μl drug was added into each pore, while control group replaced serum-free medium. Add 20 μl MTT to each hole, and then 150 μl DMSO after 4 h at 37 °C, shake for 30 min. Measure the optical density (OD) at 490 nm with enzyme standard meter.

### Combination index

On the basis of the IC-50 values of SKOV-3/DDP by nab-P and AP, the data map of Fa-Cl plot established by compusyn (version 2.0) software was used to analyze the combination of drugs. Synergism (Cl < 1): greater than expected additive effect. Additive effect (Cl = 1): the combined effect predicted by the mass-action law principle in the absence of synergism or antagonism. Antagonism (Cl > 1): small than expected additive effect.

### Western blot assay

Total cellular protein was extracted with RIPA lysate buffer (Boster Biological Technology) containing protease inhibitor and phosphorylase inhibitor (Boster Biological Technology), and determined protein concentration with BCA protein detection kit (Boster Biological Technology), then separated by SDS-PAGE electrophoresis kit (cwbiotech). The amount of each group proteins was 20μg. After separation, the proteins were transferred to PVDF membrane (0.22um). When sealed by 0.5% non-fat milk powder still 1 h, the PVDF membrane was incubated with polyclonal primary antibody and secondary antibody combined with HRP. The membrane was colored by ECL enhanced chemiluminescence kit (Boster Biological Technology) and formed by Biological Spectrum Image System Scanning.

Primary antibodies used in this study include anti-β-actin(1:5000, AP0060, Bioworld Technology, Inc), anti-bcl-2(1:1000, AF6139, Affinity), anti-Bax(1:1000, AF0120, Affinity), anti-p-VEGFR-2(1:500, AF3279, Affinity), anti-MMP-2(1:500, AF5330, Affinity). The secondary antibodies include HRP-conjugated affinipure goat anti-Rabbit IgG(1:5000, Boster Biological Technology, BA1054).

### Immunofluorescence

SKOV-3/DDP different groups were inoculated in 6 well cell cultrue cluster. A slide was placed in each hole for cell climbing. The inoculation amount of each hole was controlled at 10^5^ cells. After the cells adhered to the wall, PBS was soaked for 3 min × 2 times. Cells were fixed with 4% paraformaldehyde and soaked with PBS. Cells were permeable with 0.5% Triton X-100 room temperature. PBS was rinsed again. The PBS was dried by absorbent paper, and then the normal goat serum blocking solution was dripped on the slide for 30 min. The absorbent paper was dried. Each slide was dripped with a sufficient amount of diluted first antibody, and put into a wet box. After incubation at 4 °C overnight, it was soaked by PBST. After absorbing the superfluous liquid, the absorbent paper dripped with CY3 labeled Goat anti rabbit IgG, incubated in a wet box at 37 °C for 1 h, and then washed with PBS. DAPI was dripped in the dark and incubated in dark for 5 min. In the dark place, absorbent paper is used to absorb the climbing liquid, and the sealing liquid containing anti fluorescence quenching agent (Boster Biological Technology) was used for sealing. Images were collected under fluorescence microscope. Follow the same steps for frozen section.

Primary antibodies used in this study include anti-bcl-2(1:200, AF6139, Affinity), anti-Bax(1:200, AF0120, Affinity), anti-p-VEGFR-2(1:200, AF3279, Affinity), anti-CD31(1:200, BS90231, Bioworld Technology), The secondary antibodies include CY3 conjugated affinipure goat anti-rabbit IgG(1:200, Boster Biological Technology, BA1032).

### Transwell invasion assay

The SKOV-3/DDP cell line was treated in RPMI 1640 medium with serum free for 24 h. Then 1 × 10^5^ cells in 100 μl medium were respectively sucked into upper chamber of transwell (8 μm pore size) with 20 μl pre-coated Matrigel (coring), 500 μl culture medium containing 20% FBS was added into the lower chamber to stimulate cell travelling. After 24 h culture at 37 °C, 5% CO_2_ incubator, transwell chambers were fixed using 4% paraformaldehyde, and then stained with 0.1% crystal violet. Cells laid on upper surface of transwell membrane were wiped using a cotton swab, while cells traveled to the lower surface of membrane were photographed under a microscope. The average transmitted cells were counted in five random fields.

### Wound healing assay

5 × 10^5^ cells were inoculated into 6 well cell cultrue cluster and maintained in incubator for 12 h–24 h until cells reached 100% confluence. Then the cell monolayer was scratched to create a gap with 100 μl pipette tip followed by PBS washing. Finally, the culture medium was changed into serum free RPMI 1640 medium. The gaps were observed and photo- graphed at 0 h, 12 h and 24 h after scratching, the area of scratches were calculated by Image J software.

### Xenograft model

The BALB/C-nu were purchased from Charles River Laboratories China, all of these were almost 5-week-old female nude mouse. This study was accomplish with the approval of the ethical committee of Provincial Cancer Hospital, Shanxi, China, and followed the institutional guideline and ethical standard. In order to establish subcutaneous transplanted OC model, 2 × 10^6^ SKOV-3/DDP cell line was injected into the right axilla of each mouse. When the axillary tumor volume of the nude mice was 200 mm3, the nude mice were randomly divided into four groups, six in each group, and the following interventions were carried out every day. a): Control group, no drug intervention, ntraperitoneal perfusion of 200 μl NS, b): Group-1, nab-P 20 mg/kg, intraperitoneal perfusion+AP 150 mg/kg, gavage administration, c): Group-2, nab-P 18 mg/kg, intraperitoneal perfusion+AP 150 mg/kg, gavage administration, d): Group-3, nab-P 16 mg/kg, intraperitoneal perfusion+AP 150 mg/kg, gavage administration. Record the diet and exercise status, and measure the tumor size axis every other day,

The xenografts were measured by caliper, and the tumor volume was calculated based on length (L) and the width (W) by the following formula: V = 1/2 × L × W^2^.

### Immunohistochemistry

The tissue was dehydrated by sucrose, then each tissue made a frozen-section, 16 μm, lined with adhesive slides. Incubated with 3% hydrogen peroxide at room temperature for 10 min, washed by PBS for 2 min × 3 times; normal goat serum was incubated at room temperature for 10 min, then sealed with appropriate proportion of diluted primary antibody, washed by PBS for 2 min × 3 times overnight at 4 °C, drip with ready to use secondary antibody, incubated at 37 °C for 30 min, washed by PBS for 2 min × 3 times, drip with fresh DAB Color developing solution: control the color developing time under the microscope, wash completely with water, re-dye by the hematoxylin solution for several seconds, wash with water, dry the color developing tablets after alcohol, seal them with neutral gum, and observe under the microscope.

### Statistical analysis

SPSS 21.0 software was used to analyze the data (Means±SD). Paired samples were analyzed by paired sample T-test, and multiple samples were analyzed by one-way analysis of variance; *P*<0.05 was statistically significant.

## Result

### Effect of nab-P and AP on SKOV-3/DDP

Before exploring the combination therapy, we examined the inhibitory effect of nab-P and AP alone on ovarian cancer cells. In order to simulate platinum-resistant OC patients, we selected platinum-resistant SKOV-3 cell line that can highly express VEGFR-2, that is SKOV-3/DDP.

First, we determined the drugs concentrations of nab-P and nab-P by half inhibition concentration (IC-50) values obtained from MTT assay. Nine concentration gradients (5 × 10^− 2^ to 5 × 10^2^ of nab-P, 10^− 1^ to 10^3^ of AP) were established to intervene for 24, 48, and 72 h respectively. The results (Fig. 1a) showed that the drugs effect on SKOV-3/DDP were obviously concentration and time dependent manner. The IC-50 values were showed in Table 1. Divided SKOV-3/DDP into 3 groups and treated with nab-P and AP according to their 48 h IC-50 values. a): Control group, no drug intervention to set the black control, b): nab-P group, nab-P 20 μmol/l, c): AP group, AP 50 μmol/l.

**Fig. 1:** Effect of nab-P and AP on SKOV-3/DDP. **a** the nab-P and AP’s half inhibition concentration to SKOV-3/DDP (24, 48 and 72 h), **b** the Bax, bcl-2, p-VEGFR-2 and MMP-2 protein expression of different groups by Western blot (WB), **c** the Bax, bcl-2, p-VEGFR-2 and MMP-2 protein expression of different groups by Immunofluorescence (IF), **d** the invasion in different groups by Transwell assay, **e** the migration in different groups by Wound healing assay. Note: *P < 0.05, **P < 0.01, medication group vs control group, △P < 0.05, △△P < 0.01, comparison of two sets of data

**Table 1:** IC-50 value of nab-P and AP on SKOV-3/DDP ($\overline{\mathrm{x}}$ ± SD)

		nab-P group	AP group
IC-50 (μmol/l)	24 h	45.53 ± 4.06	65.74 ± 8.33
	48 h	20.88 ± 2.99	50.66 ± 4.96
	72 h	8.77 ± 0.64	39.54 ± 6.62

The Bax and bcl-2 are the most commonly used proteins to detect apoptosis, SKOV-3 is ovarian cancer cell line with high expression of VEGFR-2, and AP can inhibit tumor angiogenesis by inhibiting the formation of p-VEGFR-2, and MMP-2 is closely related to the ability of invasion of tumor cell. So we used Western blot (WB) and Immunofluorescence (IF) to detect the expression of Bax, bcl-2, p-VEGFR-2 and MMP-2, and Image J software was used to analyze (Fig. 1b, c). The results were showed in Table 2. The difference between Control group and medication groups were all statistically significant (*P* < 0.01). Meanwhile, the inhibition effect of nab-P and AP on the invasion of SKOV-3/DDP were verified by Transwell and Cell scratch tests (Fig. 1d, e). The results also showed in Table 2. Compared with Control group, the difference were statistically significant (*P* < 0.01).

**Table 2:** The results of WB, IF, Transwell and Would healing assay ($\overline{\mathrm{x}}$ ± SD)

		Control group	nab-P group	AP group
WB (relative gray value)	Bax	0.04 ± 0.01	0.13 ± 0.07	0.14 ± 0.09
	bcl-2	0.26 ± 0.01	0.09 ± 0.01	0.09 ± 0.01
	p-VEGFR-2	0.14 ± 0.04	0.14 ± 0.06	0.04 ± 0.01
	MMP-2	0.14 ± 0.01	0.04 ± 0.01	0.05 ± 0.01
IF (positive rate%)	Bax	2.01% ± 0.39	13.87% ± 1.91**	14.17% ± 1.69**
	bcl-2	23.9% ± 1.04	13.87% ± 2.45**	15.67% ± 1.31**
	p-VEGFR-2	25.17% ± 0.97	25.8% ± 1.94	7.4% ± 0.88**
	MMP-2	19.3% ± 1.16	10.4% ± 0.85**	10.83% ± 1.92**
Transwell (invasion cellular amount)		389 ± 25.8	41 ± 7.6**	53 ± 4.7**
Wound healing (Area recovery%)	12 h	63.54% ± 3.64	−3.89% ± 0.51**	−9.85% ± 0.62**
	24 h	84.88% ± 1.75	1.76% ± 0.12**	−5.87% ± 0.62**

Note: ** *P* < 0.01, medication group vs control group

### Effects of different doses of nab-P combined with AP on SKOV-3/DDP

From what is said above, we can draw a conclusion that for SKOV-3/DDP, both nab-P and AP can exert satisfactory anti-tumor effects alone. However, the concentration of drugs is relatively high, so we envision whether the combination of two drugs can reduce the doses of drugs and achieve the anti-tumor effect of 1 + 1 > 2. We designed the following experiments. We used a fixed concentration ratio of nab-P: AP = 1:2 to act on SKOV-3/DDP.

MTT assay detecting the IC-50 value was nab-P 5.28 μmol/l + AP 10.56 μmol/l (48 h) (Fig. 2a), the combined inhibition index (CL) was all belowed 1(Fig. 2b), that men nab-P combined with AP on SKOV-3/DDP had synergistic effect. In clinic, side effects caused by chemotherapeutic agents are often positively correlated with drug dosage. Therefore, we proposed whether the dose of nab-P could be appropriately reduced after the combination of AP without affecting the anti-tumor effect. We designed the following groups, a): Control group, no drug intervention to set the black group; b): Group-1, nab-P 5 μmol/l + AP 10 μmol/l; c): Group-2, nab-P 4.5 μmol/l + AP 10 μmol/l; d): Group-3, nab-P 4 μmol/l + AP 10 μmol/l, in which the drug dose of Group-1 was formulated according to the MTT, and the drug concentration of nab-P in Group-2 and Group-3 decreased with 0.5 μmol/l in turn. At the same time, designing e): nab-P group: nab-P 5 μmol/l and f): AP 10 μmol/l as the drug control group for comparison.

**Fig. 2:** Effects of different doses of nab-P combined with AP on SKOV-3/DDP. **a** the nab-P combined with AP’s half inhibition concentration to SKOV-3/DDP (24, 48 and 72 h), **b** Combined inhibition index, **c** the Bax, bcl-2, p-VEGFR-2 and MMP-2 protein expression of different groups by Western blot (WB), **d** the Bax, bcl-2, p-VEGFR-2 and MMP-2 protein expression of different groups by Immunofluorescence (IF), **e** the invasion in different groups by Transwell assay, **f** the migration in different groups by Wound healing assay. Note: *P < 0.05, **P < 0.01, medication group vs control group, △*P* < 0.05, △△*P* < 0.01, comparison of two sets of data

The expression of Bax, bcl-2, p-VEGFR-2 and MMP-2 in SKOV-3/DDP were also detected by WB and IF (Fig. 2c, d). The inhibition effect of nab-P combining with AP on the invasion were also verified by Transwell and Cell scratch tests (Fig. 2e, f). Compared with the Control group, the difference was obviously significant (*P* < 0.01). And there still were no significant difference between the three medication groups. In addition, there were significant differences in apoptosis, invasion and angiogenesis between nab-P and AP alone group and Group-1.

The results showed that reducing dose of nab-P had no significant effect on the anti-tumor activity when combined with AP, the results were showed as Table 3.

**Table 3:** The results of WB, IF, Transwell and Would healing assay ($\overline{\mathrm{x}}$ ± SD)

		Control group	Group-1	Group-2	Group-3	nab-P	AP
WB (relative gray value)	Bax	0.03 ± 0.00	0.15 ± 0.01**	0.14 ± 0.01**	0.14 ± 0.01**	0.10 ± 0.02**	0.09 ± 0.00**
	bcl-2	0.24 ± 0.01	0.06 ± 0.01**	0.06 ± 0.01**	0.06 ± 0.01**	0.18 ± 0.01**	0.19 ± 0.02**
	p-VEGFR-2	0.14 ± 0.01	0.03 ± 0.00**	0.04 ± 0.00**	0.04 ± 0.00**	0.13 ± 0.01	0.09 ± 0.00**
	MMP-2	0.16 ± 0.01	0.03 ± 0.00**	0.04 ± 0.00**	0.04 ± 0.00**	0.09 ± 0.01**	0.09 ± 0.00**
IF (positive rate%)	Bax	2.7% ± 0.29	23.07% ± 1.13**	21.57% ± 0.67**	21.8% ± 1.8**	12.4% ± 1.07**	10.57% ± 0.68**
	bcl-2	25.7% ± 0.65	7.57% ± 1.11**	7.4% ± 1.1**	8.2% ± 1.2**	13.33% ± 1.96**	13.73% ± 0.71**
	p-VEGFR-2	27.8% ± 0.86	6.8% ± 1.51**	7.5% ± 0.94**	8.4% ± 0.88**	24.47% ± 2.27	17.7% ± 0.52**
	MMP-2	27.1% ± 1.7	7.97% ± 1.2**	9.83% ± 1.01**	11.13% ± 0.4**	21.07% ± 1.14**	22.27% ± 0.97**
Transwell (invasion cellular amount)		391 ± 21.7	6 ± 1.3**	12 ± 2.6**	14 ± 1.9**	197 ± 29.9**	216 ± 26.1**
Wound healing (Area recovery%)	12 h	63.54 ± 4.48	−6.56 ± 0.39**	−5.28 ± 0.53**	−4.5 ± 0.39**	1.03 ± 0.05**	−2.46 ± 0.27**
	24 h	84.88 ± 2.15	−14.8 ± 0.7**	−14.37 ± 0.73**	−14.15 ± 0.61**	1.51 ± 0.07**	−2.51 ± 1.18**

Note: ** *P* < 0.01, medication group vs control group

### Effects of different doses of nab-P combined with AP on xenograft models

Through the above two parts of the experiment, we can get that nab-P combined with AP can significantly inhibit tumor growth and promote apoptosis of SKOV-3/DDP. When the dosage of nab-P is properly reduced, it can still achieve satisfactory anti-tumor effect. Therefore, at the cellular level, nab-P can reduce the dosage when combined with AP. We go further to design in vivo experiments to verify whether the results are consistent with those of in vitro.

After the establishment of xenograft models, the tumor volumes were recorded every other day (Fig. 3a), and the results as showed in Table 4. We found that there was no significant difference in tumor volume between the three medication groups, but there was between Control group(*P* < 0.01).

**Fig. 3:** Effects of different doses of nab-P combined with AP on BALB/c. **a** Growth curve of subcutaneous tumor in four groups of mice, 0 d repressed the first day of drug intervention, **b** mice and volume of tumor after exfoliation, **c** the Bax, bcl-2, CD31, p-VEGFR-2 and MMP-2 protein expression of different groups by Western blot, **d** the Bax, bcl-2, CD31, p-VEGFR-2 and MMP-2 protein expression of different groups by Immunofluorescence (400x), **e** the Bax, bcl-2, CD31, p-VEGFR-2 and MMP-2 protein expression of different groups by Immunohistochemistry (400x). Note: *P < 0.05, **P < 0.01, medication group vs control group, △*P* < 0.05, △△*P* < 0.01, comparison of two sets of data

**Table 4:** Changes of tumor volume before and after administration in different groups ($\overline{\mathrm{x}}$ ± SD)

Tumor volumes (mm^3^)	Drug-before	Drug-after
Control group	234.83 ± 28	1452.83 ± 61.47
Group-1	230.17 ± 31.66	144 ± 37.65**
Group-2	224.83 ± 28	142.33 ± 31.4**
Group-3	233.67 ± 29.37	138.83 ± 31.43**

Note: ** *P* < 0.01, medication group vs control group

We also analyzed the expression of related proteins in tumor masses by WB, IF and immunohistochemistry (IHC) (Fig. 3c, d, e). The three medication groups were had no difference between them, while compare with Control group, there were all significant difference(*P* < 0.01). The WB’s relative gray value and IF, IHC ‘s positive rate(%) as Table 5.

**Table 5:** The results of WB, IF, IHC ($\overline{\mathrm{x}}$ ± SD)

		Control group	Group-1	Group-2	Group-3
WB (relative gray value)	Bax	0.08 ± 0.02	0.18 ± 0.12**	0.17 ± 0.17**	0.17 ± 0.02**
	bcl-2	0.17 ± 0.02	0.07 ± 0.01**	0.09 ± 0.01**	0.09 ± 0.01**
	CD31	0.75 ± 0.04	0.16 ± 0.02**	0.16 ± 0.04**	0.2 ± 0.01**
	p-VEGFR-2	0.26 ± 0.02	0.16 ± 0.03**	0.18 ± 0.01**	0.19 ± 0.01**
	MMP-2	0.71 ± 0.02	0.29 ± 0.03**	0.3 ± 0.02**	0.29 ± 0.01**
IF (positive rate%)	Bax	3.37% ± 0.91	20.97 ± 2.09**	19.13 ± 2.78**	19.73 ± 1.52**
	bcl-2	17.17 ± 1.69	3.23 ± 1.35**	2.43 ± 0.79**	2.57 ± 0.5**
	CD31	24.1 ± 1.15	6.73 ± 1.47**	9.53 ± 1.6**	9.7 ± 1.96**
	p-VEGFR-2	16.77 ± 1.03	3.0 ± 0.29**	3.83 ± 0.61**	4.07 ± 1.04**
	MMP-2	13.2 ± 1.53	2.77 ± 0.54**	2.87 ± 0.49**	2.93 ± 0.69**
IHC (positive rate%)	Bax	13.2% ± 1.07	34.17 ± 1.11**	32.83 ± 0.95**	32.77 ± 1.16**
	bcl-2	31.73 ± 1.67	13.33 ± 1.59**	14.63 ± 1.48**	13.87 ± 1.89**
	CD31	36.1 ± 1.69	11.63 ± 1.2**	12.67 ± 1.52**	12.33 ± 2.24**
	p-VEGFR-2	35.47 ± 2.93	17.1 ± 1.31**	17.53 ± 1.6**8	18.23 ± 1.25**
	MMP-2	34.9 ± 2.38	14.53 ± 1.17**	15.27 ± 0.74**	15.57 ± 2.75**

Note: ** *P* < 0.01, medication group vs control group

During the experiment, by observing the quality of life of the mice, we found that after the intervention of nab-P and AP, the majority side effects in the medication groups were anorexia and decreased activity. Therefore, we evaluated the quality of life of different groups by average amount of daily diet and 1 h activity (Table 6). There is no apparent difference of the quality of life in the 4 groups before the treatment. When AP combined with different doses of nab-P, the quality of life was negatively correlated with the dose of nab-P. The difference of two evaluation indexes between the each experimental groups and the control group were statistically significant (P < 0.01).

**Table 6:** Effects of different doses of nab-P combined with AP on the quality of life of mice

Group	Total (n)	Average amount of daily diet(g)			One hour activity (min)		
		Before medication	After medication	P	Before medication	After medication	P
Control group	6	6.79 ± 0.21	6.90 ± 0.19	0.64	18.63 ± 0.15	19.35 ± 0.14	0.62
Group-1	6	6.78 ± 0.21	4.50 ± 0.17**	< 0.01	17.54 ± 0.15	6.11 ± 0.16**	< 0.01
Group-2	6	6.91 ± 0.19	5.64 ± 0.15**	< 0.01	17.68 ± 0.15	6.29 ± 0.12**	< 0.01
Group-3	6	6.62 ± 0.16	5.55 ± 0.13**	< 0.01	17.95 ± 0.14	6.34 ± 0.13**	< 0.01

Note: Average daily intake represents the average food consumption of mice in the two stages (Before and After medication, Control group was replaced by NS), One hour activity expresses activity time of mice within one hour from 9:00 to 10:00 and 21:00 to 22:00, **P < 0.01, medication group vs control group

## Discussion

Although the therapeutic technologies for ovarian cancer continues to improve, the mortality rate remains high [21], especially for patients with recurrent epithelial ovarian cancer. More importantly, the long-term use of chemotherapeutics will damage the normal tissues of patients, result in drug resistance in patients, even the failure of clinical treatment [22]. In this experiment, we tested the targeting drug AP in combination with several different doses chemotherapeutics nab-P against SKOV-3/DDP. And results showed that both nab-P and AP can play satisfactory anti-tumor effects against platinum-resistant ovarian cancer cells, and when combined, their respective anti-tumor effects are enhanced. Furthermore, when combined with AP, if nab-P properly reduced, the two drugs can still achieve ideal anti-tumor effect.

The following will elaborate.

Firstly, we analyzed the drug effects of nab-P and AP alone at the cellular level. We obtained the IC-50 value of nab-P and AP to SKOV-3/DDP. The results showed that IC-50 of nab-P was lower than AP, this indicated that the drug effect of nab-P on SKOV-3/DDP is slightly stronger. Apoptosis is a form of cell death, which plays an important role in maintaining the balance between normal cell death and cell division [23]. Inhibition of apoptosis and abnormal cell proliferation and differentiation are the biological basis of tumorigenesis [24]. And promoting apoptosis of tumor cells is one of the most important methods in tumor therapy [25]. The proteins of Bax and bcl-2 are key in regulating apoptosis. Therefore, we used WB and IF to analyze the effect of treated on the expression of these two proteins. The results showed after nab-P and AP intervention, the expression of Bax was higher than Control group, bcl-2 contrary. That’s means that both nab-P and AP can promote apoptosis of SKOV-3/DDP. Tumor growth mainly depends on tumor angiogenesis [26], and vascular endothelial growth factor (VEGF) is an important factor in the latter. Distributing widely in normal and tumor tissues, it can stimulate the proliferation, survival and migration of endothelial cells through the corresponding cell surface receptors and signal pathways, which is one of the important factors for the growth and survival of endothelial cells [27]. VEGFR is the main functional receptor of VEGF, and its subtype, VEGFR-2, is considered to be a key molecule in the VEGF signaling pathway that induces angiogenesis. So, inhibiting the binding of VEGFR-2 to VEGF or the transmission of its downstream signaling pathways all can achieve the purpose of inhibiting tumor angiogenesis and then tumor growth [28]. Targeting drug Apatinib can specifically act at the ATP binding site of VEGFR-2, inhibiting the production of p-VEGFR-2 and blocking downstream signal transduction pathways. Therefore, we tested expression of p-VEGFR-2 in different groups. The results also confirmed that in AP group, the expression of p-VEGFR-2 was reduction, while there was no significant difference between nab-P group and control group. Several studies have shown that matrix metalloproteinases play an important role in tumor cell invasion and metastasis [29], while MMP-2 is an important component [30]. In medication groups, the expression of MMP-2 were declined when compared with Control group. We also used Transwell and Cell scratch test to verify the changes of invasion and migration of SKOV-3/DDP in different groups. As the same as the expected results, after the intervention of nab-P and AP, the invasive ability of cells in vitro and healing rate decreased significantly. Therefore, we can draw the first conclusion that nab-P and AP can play a good anti-tumor effect on SKOV-3/DDP. The results are the same with Jing, Momeny, Tipton et al. [31–33]

However, considering the limitation of single drug therapy, combination therapy is a routine means for clinical tumor treatment [34]. In recent years, the combination of chemotherapeutics and targeted drugs has made significant breakthroughs in both basic research and clinical application of OC [19, 35, 36]. nab-P is a kind of paclitaxel wrapped by human albumin, which can enter the tumor cells easily, increase the drug concentration in tumor cells, and achieve ideal therapeutic effect on OC. Nevertheless, once the tumor burden is reduced after nab-P treatment, it may lead to increased reactivity of VEGF signaling pathway expression [37]. If some inhibitor about VEGF is used at the same time, the expression of VEGF and its related proteins will be continuously inhibited, tumor angigogenesis will be reduced simultaneously, so as to achieve better anti-tumor effect, AP is such one. So we expect the combination of these two drugs to be more effective.

According to above-mentioned analytical results, we designed the second part of the experiment. We also tested the inhibitory effect of nab-P combined AP on SKOV-3/DDP by MTT assay, and with the help of compusyn (version 2.0) software analysised the Cl of the two drugs. The results showed that, after nab-P combined with AP, it had a strong inhibitory effect on SKOV-3/DDP, and played a synergistic effect. On the basis of IC-50 value, we set up the different concentration of nab-P combined with AP as combination groups, and the same dose of nab-P and AP single drug as drug control groups to explore the improvement effect of anti-tumor and the influence of different doses of nab-P on the efficacy. Western blot and immunofluorescence experiments also be used to observe the expression of related proteins (Bax, bcl-2, p-VEGFR-2 and MMP-2). According to the results, after combined with AP, appropriate reduction of nab-P did not affect the anti-tumor effect of both drugs, while compared with nab-P and AP single drug group, the difference were statistically significant. Transwell and Cell scratch test’s results also showed the combination of drugs greatly weakened the invasion and migration of SKOV-3/DDP. Above that, we can obtain another conclusion that at the cellular level, when nab-P and AP are used in combination, the idea of reducing drug toxicity by reducing the amount of nab-P is feasible.

After obtaining satisfactory results at the cell level, we designed animal experiments to verify whether the results of the combination drugs at the animal level are consistent with those at the cell. This is also the third part of the experiment. Different concentration of nab-P were combined with the same dose of AP. The shrinkage of tumor mass were observed by calculating the volume of subcutaneous tumor in mice after administration. The results showed that after the combination treatment, the tumor volume decreased significantly, and there was no significant difference among the three combination groups. In addition, Western blot, immunofluorescence and immunohistochemistry were carried out to detect the related proteins. The results showed that the expression of bcl-2, CD31, p-VEGFR-2, MMP-2 all decreased significantly while Bax increased, compared with the control group, the difference was statistically significant, but there were no obvious difference among the three combination groups, which was highly consistent with the experimental results at the cell level. The side effects caused by chemotherapy drugs are important factors affecting the quality of life of patients [38]. In order to verify the effect of reducing the doses of nab-P on the survival of nude mice, we set up two observation indexes: average amount of daily diet and one hour exercise. We found that there was a significant negative correlation between the quality of life of mice and the dosage of nab-P. Therefore, we can draw the third conclusion, that is, in vivo experiments, after nab-P combined with AP, appropriate reduction of the recommended dosage of nab-P can achieve the purpose of reducing the adverse reactions in mice.

In a word, in this experiment, we combined the targeting drug AP with the chemotherapy drug nab-P to act on the SKOV-3/DDP and xenograft models, and found that the combination of the two drugs can significantly inhibit the proliferation and invasion of the tumor. Secondly, after the combination, it can be properly reduced the doses of nab-P without effecting the anti-tumor effects. This suggests that, in the clinical treatment, the scheme of combination can bring less side effects.

Due to the certain toxicity of chemotherapy drugs, patients are prone to some adverse reactions such as myelosuppression, gastrointestinal reactions, etc. Therefore, if the combination can reduce the dosage of nab-P on the basis of not reducing the therapeutic effect, and the adverse reactions will be correspondingly reduced, which may improve the quality of life of patients.

## Data Availability

The datasets used and analysed during the current study are available from the corresponding author (Rong Li) on reasonable request.

## Abbreviations

OC: Ovarian cancer
NCCN: The National Comprehensive Cancer Network
PFS: Progression-free survival
nab-P: Paclitaxel (aluminum binding type)
AP: Apatinib
TK: Tyrosine kinase
TKI: Tyrosine kinase inhibitors
VEGFR-2: Vascular endothelial growth factor receptor-2
ORR: Objective response rate
VEGF: Vascular endothelial growth facto
Cl: Combination index
